# Long Noncoding RNA H19 Derived from M2 Tumor-Associated Macrophages Promotes Bladder Cell Autophagy via Stabilizing ULK1

**DOI:** 10.1155/2022/3465459

**Published:** 2022-05-14

**Authors:** Yuanyuan Guo, Wei Sun, Wuyue Gao, Liqiang Li, Yujie Liang, Zhijie Mei, Beibei Liu, Rui Wang

**Affiliations:** ^1^Department of Urology, The First Affiliated Hospital of Bengbu Medical College, Bengbu, Anhui 233004, China; ^2^Department of Oncology, The First Affiliated Hospital of Bengbu Medical College, Bengbu, Anhui 233004, China

## Abstract

**Purpose:**

M2-like tumor-associated macrophages (TAMs) are crucial component of immune infiltration in tumor microenvironment (TME), and exosomes derived from TAMs contributed to the regulation of tumor progression through cellular communication. However, in bladder cancer, the role of exosomal components still remains largely unknown. In the current study, we investigated the role of exosomes derived from M2-like TAMs in the regulation of autophagy in bladder cancer (BC) cells.

**Methods:**

THP-1 cells were stimulated with IL-4 and IL-13 for the polarization of TAMs, and exosomes were extracted by ultracentrifugation. H19 overexpression plasmid and H19 siRNAs were used in the study. Fluorescent analysis was performed for GFP-LC3 detection. Levels of autophagy and potential target were confirmed by western blot assay and immunoprecipitation.

**Results:**

We found that TAMs-exosome treatment significantly enhanced autophagy in BC cells, and the expression of lncRNA H19 was greatly upregulated in TAMs-exosome. Silencing of lncRNA H19 in TAMs-exo obviously decreased the levels of LC3-II expression whereas the p62 levels were increased. Mechanistically, silencing of exosomal H19 from TAMs alleviated ULK1 stabilization in BC cells through promoting K48-linked polyubiquitination of ULK1. At last, we found that overexpression of exosomal H19 from TAMs suppressed the interaction between ULK1 and its specific E3 ligase NEDD4L in BC cells.

**Conclusion:**

We revealed the effect of TAMs-exo-contained lncRNA H19 on regulating autophagy of bladder cancer cells, which indicated that targeting TAMs-H19 is a promising therapeutic strategy for the treatment of BC.

## 1. Introduction

Bladder cancer (BC) is characterized by multiple lesions and high postoperative recurrence rate, which poses challenges for the treatment of bladder cancer [1, 2]. With increasing understanding of the molecular mechanisms underlying the pathogenesis of bladder cancer, it has been found that proliferation, apoptosis, migration, angiogenesis, and other processes are essential for cancer development; however, the precise molecular mechanisms of BC progression still remain largely unknown [3].

Recently, autophagy has been proved to play critical roles in almost all the diseases especially in cancers [4, 5]. During BC development and tumorigenesis, autophagy was found to act as a double-edged sword in respect of molecular mechanisms of bladder cancer [6]. Therefore, a further understanding of the mechanism by which autophagy plays in bladder cancer is essential for the corresponding treatment of bladder cancer.

Tumor cells and various stromal cells, immune cells, and cytokines constitute a complex tumor microenvironment (TME). Among them, tumor-associated macrophages (TAMs) are one of the most important stromal cells, which actively participate in the process of tumor genesis, growth, infiltration, and metastasis [7]. It has been reported that CXCL1-mediated interaction of cancer cells with TAMs and cancer-associated fibroblasts (CAFs) promotes tumor progression in BC [8]. BMP4 secreted by bladder cancer cells was found to be contributed to M2 macrophage polarization and aggravated tumor metastasis [9]. Therefore, extended studies on TAMs could provide novel and effective ways for BC treatment.

In the current study, we found that exosomal lncRNA H19 from TAMs positively correlated with the regulation of autophagy status in BC cells. Mechanistically, we found that TAMs-exo-contained H19 interrupted the interaction between autophagy-promoting protein Unc-51 such as autophagy-activating kinase 1 (ULK1) and its specific E3 ligase NEDD4-like E3 ubiquitin protein ligase (NEDD4L), therefore promoting ULK1 stabilization-induced abnormal activation of autophagy in BC cells, and our findings suggested exosomal lncRNA H19 derived from TAMs as a potential target for the treatment of BC.

## 2. Materials and Methods

### 2.1. Cell Culture and M2-Like TAM Polarization

Human monocyte cell line THP-1 and human bladder cancer cell lines T24 and HTB-1 were purchased from the Chinese Academy of Sciences (Shanghai, China) and cultured in DMEM with the existence of 10% FBS (Gibco), 100 U/ml penicillin, and 100 *µ*g/ml streptomycin. The cells were grown at 37°C, 5% CO_2_ condition. For M2-like TAM polarization, 20 ng/ml IL-4 and IL-13 (R&D Systems) was administered for 24 hours to induce M0-M2 polarization as described previously [10].

### 2.2. Exosome Isolation and Identification

Exosome isolation was performed as reported previously [11]. In brief, after macrophage polarization, the culture medium was changed to exosome-depleted culture medium. 24 hours later, the supernatants were collected and centrifuged at 2000 ×g for 20 min, filtered through a 0.22 *μ*m filter, and ultracentrifuged at 100,000 ×g for 1.5 hours. Pelleted vesicles were washed with PBS and centrifuged again at 100,000 ×g for 1.5 hours to obtain exosomes. Transmission electron microscopy (TEM) and Nano-LC-MS/MS analysis were performed to identify exosomes as described [12].

### 2.3. Fluorescent Observation

T24 cells were transfected with the GFP-LC3 plasmid for 24 hours, followed by the incubation of exosomes from THP-1 or TAMs. LC3 puncta and LC3 expression were detected by a fluorescence microscope after starvation for 4 h.

### 2.4. Plasmids and siRNAs

The plasmids for lncRNA H19 overexpression and GFP-LC3 were purchased from MDL Biotechnology (Beijing, China), and the synthesized scrambled siRNA and H19 siRNA were purchased from Thermo Fisher. Lipofectamine 2000 (Invitrogen, Carlsbad, CA, USA) and Lipofectamine RNAiMAX (Invitrogen, Carlsbad, CA, USA) were used to transfect plasmids or siRNAs into cells according to the manufacturer's protocol.

### 2.5. Quantitative Real-Time PCR (qRT-PCR)

TRIzol reagent (Invitrogen, Carlsbad, CA, USA) was used to extract the total RNAs in cells according to the manufacturer's instruction. For reverse transcription, the PrimeScriptTM RT reagent kit (TaKaRa, Dalian, China) was applied to obtain the first-strand complementary DNA. Quantitative PCR was examined by SYBR Green PCR Master Mix (TaKaRa, Dalian, China) according to the manufacturer's instruction. Cycle conditions were used as follows: 95.0°C for 5 mins and 40 cycles at 95.0°C for 30 s and 70.0°C for 60 s, and final extension at 70.0°C for 7 mins. Quantifications were performed by a comparative method (2-DDCt) using GAPDH transcripts as an internal control. The sequences for the primers were shown as follows: lncRNA H19: forward: 5′-CAC TGG CCT CCA GAG CCC GT-3′ and reverse: 5′-CGT CTT GGC CTT CGG CAG CTG-3′ and GAPDH: forward: 5′-CTG GGC TAC ACT GAG CAC C-3′ and reverse: 5′-AAG TGG TCG TTG AGG GCA ATG-3′.

### 2.6. Western Blot Assay and Immunoprecipitation (IP)

Western blot and immunoprecipitation analysis were performed as described previously [13]. The antibodies for GAPDH (sc-47724; 1 : 1000), p62 (sc-101542; 1 : 1000), anti-LC3 (sc-398822; 1 : 1000), and individual secondary antibodies were purchased from Santa Cruz (Santa Cruz Biotechnology, Santa Cruz, CA). The antibodies for ATG5 (#12994; 1 : 1000), ATG13 (#13468; 1 : 1000), ULK1 (#8054; 1 : 1000), and NEDD4L (#4013; 1 : 1000) were all obtained from Cell Signaling Technology (Cell Signaling Technology Inc., Beverly, USA).

### 2.7. Xenografted Tumors

BALB/c nude mice (five to six weeks old, purchased from Vital River, Beijing, China) were used to establish xenograft model (five mice per group). All animal procedures were in compliance with the National Institutes of Health (NIH) Guidelines for the Care and Use of Experimental Animals, and the models were approved by the Animal Ethics Committee of Bengbu Medical College. T24 cells (2 × 10^6^) were subcutaneously injected into the flank of the nude mice, and 6 days later when mice had palpable tumors, TAMs were transfected with si-Control or si-H19, and the exosomes were collected (10 *μ*g) and injected into the center of the xenograft tumor tissues every three days. A Vernier calliper was used to monitor the volume of tumors every 6 days (volume = width^2^ × length × 1/2). At day 30, the mice were euthanized and sacrificed and the tumors were resected.

### 2.8. Statistical Analysis

Data were expressed as the mean ± SD of three experiments in the study. Student's *t*-test was used to determine the statistical significance between the two groups. *p* < 0.05 was considered statistically significant.

## 3. Results

### 3.1. M2-TAM-Derived Exosomes Promote Autophagy in Bladder Cancer Cells

At first, we isolated the exosomes from M0 and TAMs, and the exosomes were identified by transmission electron microscopy (TEM) (Figure 1(a)), Nano-LC-MS/MS analysis (Figure 1(b)), and western blot analysis of exosome marker proteins (CD9, CD81, and HSP70) (Figure 1(c)). As shown in Figure 1(d), the autophagy marker LC3-II significantly increased and another marker p62 expression was decreased in both T24 and HTB-1 BC cells after TAMs-exosome treatment. In addition, the late-stage autophagy inhibitor Bafilomycin A1 (Baf A1) was used to block the fusion of autophagosomes with lysosomes, and in the presence of Baf A1, the accumulation of LC3-II was greatly enhanced in T24 cells administered with TAMs-exo, which indicated the increase of the autophagic flux (Figure 1(e)). Furthermore, we detected the effect of TAMs-exo on autophagosome formation in GFP-LC3-transfected T24 cells, and we found that TAMs-exo treatment significantly enhanced the expression and puncta number of GFP-LC3 (Figures 1(f) and 1(g)).

### 3.2. lncRNA H19 Expression Is Upregulated in Exosomes from TAMs

In order to illustrate the role of lncRNA H19 in TAMs-exo-induced BC cell autophagy, we examined the expression of lncRNA H19 in T24, HTB-1, M0 THP-1, and TAMs at first. As shown in Figure 2, the expression of lncRNA H19 was significantly enhanced in TAMs compared with other cells. Furthermore, we detected the expression of lncRNA H19 in TAMs-exo or M0-exo, and we found that the expression of H19 dramatically increased in TAMs-exosomes (Figure 2(b)). Moreover, we detected whether exosomal lncRNA H19 could be taken up by BC cells, and we found that high expression levels of H19 were observed in TAMs-exo-treated BC cells, which indicated that lncRNA H19 was transferred from TAMs-exosome into BC cells.

### 3.3. Silencing of H19 in TAMs-Exo Inhibits Autophagy in Bladder Cancer Cells

We silenced lncRNA H19 in TAMs, and the secreted expression of lncRNA H19 in TAMs exosomes was examined by qRT-PCR, and the efficiency of H19 silencing was confirmed as shown in Figure 3(a). Moreover, we detected the role of lncRNA H19 in BC autophagy. We found that silenced H19 in TAMs-exo obviously increased the expression of p62 in T24 and HTB-1 cells (Figure 3(b)); in addition, LC3-II levels were suppressed by H19-silenced TAMs-exo-treated BC cells (Figure 3(b)). Furthermore, Baf A1 administration confirmed that silencing of TAMs-exo decreased the autophagic flux in T24 cells (Figure 3(c)). Consistent results of LC3-positive cells are shown in Figures 3(d) and 3(e).

### 3.4. Overexpression of H19 in TAMs-Exo Promotes Autophagy in Bladder Cancer Cells

We also overexpressed lncRNA H19 in TAMs, and the overexpression efficiency of H19 in TAMs-exo was examined as shown in Figure 4(a). We found that overexpression of H19 in TAMs-exo significantly increased the expression of LC3-II and inhibited p62 expression in BC cells (Figure 4(b)). Furthermore, we observed that H19-overexpressed TAMs-exo treatment enhanced LC3-II expression in the presence of Baf A1 which aggravated the autophagic flux (Figure 4(c)). Consistent with the silencing results, H19-overexpressed TAMs-exo dramatically increased the expression and puncta formation of GFP-LC3 (Figures 4(d) and 4(e)).

### 3.5. TAMs-Exo-Derived lncRNA H19 Stabilized ULK1 in Bladder Cancer Cells

To explore the precise mechanisms about lncRNA H19-regulated autophagy, we detected the levels of several critical adaptors of autophagy including ULK1, ATG13, and ATG5. We observed that the expression of ATG13 and ATG5 was not affected by H19-silenced TAMs-exo administration in both T24 and HTB-1 cells (Figure 5(a)) whereas the ULK1 levels were significantly downregulated by H19-silenced TAMs-exo treatment (Figure 5(a)). Consistently, we found that overexpression of lncRNA H19 in exosomes from TAMs obviously increased the expression of ULK1 in BC cells, but had no effect on ATG13 and ATG5 expression (Figure 5(b)). Furthermore, we used cycloheximide (CHX) to interrupt the protein synthesis and monitored the degradation of ULK1, and more rapid degradation of ULK1 was observed in H19-silenced TAMs-exo-treated T24 cells (Figures 5(c) and 5(d)). In addition, we examined whether ULK1 polyubiquitination levels were affected by exosomal H19, and we found that silencing of H19 in TAMs-exo dramatically increased the levels of K48-linked polyubiquitination in the existence of the proteasome inhibitor mg132 (Figure 5(e)).

### 3.6. TAMs-Exo-Derived lncRNA H19 Prevents Interaction between ULK1 and NEDD4L in Bladder Cancer Cells

It was previously reported that K48-linked polyubiquitination levels of ULK1 could be modified by E3 ligase NEDD4L [14], we examined whether exosomal H19-induced decreased K48-ubiquitination was related to the NEDD4L interaction with ULK1. Interestingly, we found that silencing of exosomal lncRNA H19 from TAMs significantly enhanced the interaction between NEDD4L and ULK1 (Figure 6(a)). Consistently, we observed that overexpression of lncRNA H19 suppressed the interaction between NEDD4L and ULK1 (Figure 6(b)).

### 3.7. TAMs-Exo-Derived lncRNA H19 Aggravates Autophagy In Vivo

Finally, we established the xenograft model to demonstrate the effect of TAMs-exo-derived H19 on tumor progression and autophagy in vivo. As shown in Figure 7(a), TAMs-exo treatment enhanced tumor progression, whereas H19-silenced TAMs-exo significantly suppressed tumor formation. Moreover, tumor volume and tumor weight were all inhibited by H19-silenced TAMs-exo administration (Figures 7(b) and 7(c)). At last, we examined the protein levels of expression of LC3-II, p62, and ULK1, and we observed that the *in vivo* results were consistent with the *in vitro* results (Figure 7(d)), which meant that H19, indeed, stabilized ULK1 to enhance autophagy.

## 4. Discussion

As far as we know, the current manuscript is the first publication which reported that exosomal lncRNA H19 promoted autophagy status in the BC cells through inhibiting interaction between NEDD4L and ULK1 and stabilization of ULK1. This study extends our understanding of the regulatory mechanism of ULK1 and suggests that H19 in tumor microenvironment could be a potential target for bladder cancer treatment.

TAMs can exert both tumor-promoting and immunosuppressive effects through multiple ways based on the secretion of various kinds of growth factors, cytokines, chemokines, and nucleotides [15, 16]. Exosome pathway is an important means of intercellular communication and plays a very crucial role in communication between tumor cells and M2-TAMs [17]. Bladder cancer cell-secreted exosomal miR-21 has been reported to activate the PI3K/AKT pathway in TAMs to promote cancer progression [18]. Conversely, M2-like TAMs-derived exosomes could facilitate HCC metastasis by transferring *α*m*β*2 integrin to tumor cells [19], and TAMs exosomal microRNA-501-3p contributes to the progression of pancreatic ductal adenocarcinoma through the TGFBR3-mediated TGF-*β* signaling pathway [20]. In the current study, we found that TAMs-exosomes significantly enhanced the autophagy of BC cells because of the increased LC3-II expression and decreased levels of p62, which suggested that the inclusions of TAMs-exosomes contained the regulatory effector of autophagy process in BC cells.

Due to the double-edged sword nature of autophagy, lncRNA-mediated autophagy also exhibited different effects on tumor progression [21]. For instance, lncRNA PVT1 promotes gemcitabine resistance of pancreatic cancer via activating the Wnt/*β*-catenin and autophagy pathway [22]. lncRNA SNHG11 promotes gastric cancer progression by activating the Wnt/*β*-catenin pathway and oncogenic autophagy [23]. In the current study, we found that lncRNA H19 was overexpressed in the exosomes derived from TAMs, and silencing of exosomal H19 in TAMs-exo significantly suppressed the autophagy process in BC cells as shown of decreased LC3-II expression and LC3 puncta formation, and consistent results were obtained in the H19-overexpressed experiments. These findings suggested that TAMs could promote the autophagy process of BC cells through transferring exosomal lncRNA H19.

Unc-51-like autophagy activating kinase 1 (ULK1) is an important component of autophagy initiation complex and plays an essential role in the initiation of autophagy [24]. Taking ULK1 as the therapeutic target, intervening and regulating autophagy is thought to provide a new direction for the treatment of BC [25]. The expression of ULK1 could be downregulated by its E3 ligase NEDD4L, leading to the proteasomal degradation of NEDD4L [26]. In the current research, we found that silencing of H19 in exosome derived from TAMs decreased the expression of ULK1 in BC cells, but the expression of ATG13 and ATG5 was not affected by H19. Alleviated ULK1 stabilization was also confirmed in the presence of CHX, and the levels of K48-linked polyubiquitination were obviously attenuated in H19-silenced TAMs-exo-treated BC cells. Mechanistically, we found that H19 suppressed the interaction between ULK1 and NEDD4L, therefore stabilizing the expression of ULK1 and promoting autophagy status.

## 5. Conclusion

In conclusion, we illustrated the high expression of lncRNA H19 in TAMs-exo and the effect of exosomal H19 on BC cell autophagy. We also revealed the potential mechanism of H19 on the regulation of autophagy and suggested lncRNA H19 as a potential medical target for the treatment of BC.

## Figures and Tables

**Figure 1:** M2-TAM-derived exosomes promote autophagy in bladder cancer cells. (a) Representative electron micrograph of exosomes derived from TAMs (scale bar, 100 nm). (b) The diameter of exosomes derived from the medium of M0 or TAMs. (c) Western blot analysis of the expression of CD9, CD81, and HSP70 in the cells and exosomes. (d) Western blot analysis of protein levels of p62 and LC3 in M0-exo or TAMs-exo-treated BC cells after starvation for 2 h. (e) Western blot analysis of protein levels of LC3 in M0-exo or TAMs-exo-treated BC cells with or without the presence of Baf A1 (0.1 *μ*M) after starvation for 2 h. (f) Fluorescence image of GFP-LC3 in M0-exo or TAMs-exo-treated BC cells after starvation for 2 h. (g) Quantification of LC3-positive cells in (c). Data shown are representative images or expressed as the mean ± SD. ^*∗∗∗*^*p* < 0.001 compared to the control.

**Figure 2:** lncRNA H19 expression is upregulated in exosomes from TAMs. (a) qRT-PCR analysis of the expression of lncRNA H19 in T24, HTB-1, M0-THP-1, and M2-TAMs. (b) qRT-PCR analysis of the expression of lncRNA H19 in exosomes derived from M0-THP-1 or M2-TAMs. (c) After incubation with exosomes derived from M0-THP-1 or M2-TAMs for 24 h, the expression of lncRNA H19 in BC cells was detected by qRT-PCR. Data shown are representative images or expressed as the mean ± SD. ^*∗∗∗*^*p* < 0.001 compared to the control.

**Figure 3:** Silencing of H19 in TAMs-exo inhibits autophagy in bladder cancer cells. (a) The efficiency of H19 siRNA was examined by qRT-PCR in TAMs-exosomes. (b) Western blot analysis of protein levels of p62 and LC3 in control or H19-silenced TAMs-exosome-treated BC cells after starvation for 2 h. (c) Western blot analysis of protein levels of p62 and LC3 in control or H19-silenced TAMs-exosome-treated BC cells with or without the presence of Baf A1 (0.1 *μ*M) after starvation for 2 h. (d) Fluorescence image of GFP-LC3 in control or H19-silenced TAMs-exosome-treated BC cells after starvation for 2 h. (e) Quantification of LC3-positive cells in (d). Data shown are representative images or expressed as the mean ± SD. ^*∗∗∗*^*p* < 0.001 compared to the control.

**Figure 4:** Overexpression of H19 in TAMs-exo promotes autophagy in bladder cancer cells. (a) The efficiency of H19 overexpression was examined by qRT-PCR in TAMs exosomes. (b) Western blot analysis of protein levels of p62 and LC3 in control or H19-overexpressed TAMs-exosome-treated BC cells after starvation for 2 h. (c) Western blot analysis of protein levels of p62 and LC3 in control or H19-overexpressed TAMs-exosome-treated BC cells with or without the presence of Baf A1 (0.1 *μ*M) after starvation for 2 h. (d) Fluorescence image of GFP-LC3 in control or H19-overexpressed TAMs-exosome-treated BC cells after starvation for 2 h. (e) Quantification of LC3-positive cells in (d). Data shown are representative images or expressed as the mean ± SD. ^*∗∗∗*^*p* < 0.001 compared to the control.

**Figure 5:** TAMs-exo-derived lncRNA H19 stabilized ULK1 in bladder cancer cells. (a) Western blot analysis of protein levels of ULK1, ATG13, and ATG5 in control or H19-silenced TAMs-exosome-treated BC cells after starvation for 2 h. (b) Western blot analysis of protein levels of ULK1, ATG13, and ATG5 in control or H19-overexpressed TAMs-exosome-treated BC cells after starvation for 2 h. (c) After treatment with the protein synthesis inhibitor CHX for indicated times, the protein levels of ULK1 in H19-silenced TAMs-exosome-treated T24 cells were examined by western blot. (d) Quantification of ULK1 expression in (c). (e) Western blot analysis of K48-ub levels of ULK1 in control or H19-silenced TAMs-exosome-treated BC cells after starvation for 2 h. Data shown are representative images or expressed as the mean ± SD. ^*∗∗*^*p* < 0.01 compared to the control.

**Figure 6:** TAMs-exo-derived lncRNA H19 prevents interaction between ULK1 and NEDD4L in bladder cancer cells. (a) Western blot analysis of interaction between ULK1 and NEDD4L in control or H19-silenced TAMs-exosome-treated BC cells after starvation for 2 h in the presence of the proteasome inhibitor mg132. (b) Western blot analysis of interaction between ULK1 and NEDD4L in control or H19-overexpressed TAMs-exosome-treated BC cells after starvation for 2 h. Data shown are representative images or expressed as the mean ± SD.

**Figure 7:** TAMs-exo-derived lncRNA H19 aggravates autophagy *in vivo*. (a) Images of representative tumors excised from mice in groups. (b, c) The volume (b) and weight (c) of xenograft tumors were measured (*N* = 5 per group). (d) Western blot results of LC3, p62, and ULK1 in tumors of groups. Data shown are representative images or expressed as the mean ± SD. ^*∗∗∗*^*p* < 0.001.

## Data Availability

All data are available from the corresponding author upon request.
